# A Dynamic Community Detection Method for Complex Networks Based on Deep Self-Coding Network

**DOI:** 10.1155/2022/7084084

**Published:** 2022-07-31

**Authors:** Yusha Zhang, Xiongliang Xiao

**Affiliations:** ^1^School of Computer Science and Engineering, Hunan University of Information Technology, Changsha 410151, Hunan, China; ^2^School of Electronic Science and Engineering, Hunan University of Information Technology, Changsha 410151, Hunan, China

## Abstract

Aiming at the problem of community detection in complex dynamic networks, a dynamic community detection method based on graph convolution neural network is proposed. An encoding-decoding mechanism is designed to reconstruct the feature information of each node in the graph. A stack of multiple graph convolutional layers is considered as an encoder that encodes the node feature information into the potential vector space, while the decoder employs a simple two-layer perceptron to reconstruct the initial node features from the encoded vector information. The encoding-decoding mechanism achieves a re-evaluation of the initial node features. Subsequently, an additional local feature reconstruction loss is added after the decoder to aid the goal of graph classification. Further, stochastic gradient descent is applied to solve the problem in the loss function. Finally, the proposed model is experimentally validated based on the Karate Club and Football datasets. The experimental results show that the proposed model improves the NMI metric by an average of 7.65% and effectively mitigates the node oversmoothing problem. The proposed model is proved to have good detection accuracy.

## 1. Introduction

With the development of information technology and the increasing popularity of network media, the network community carries the self-information of massive data objects and the relationship between them [1]. How to divide the subnetworks of complex networks in biology, communication, finance, and other fields according to the network structure and node characteristics, to realize accurate community detection and further complete the effective mathematical modeling, evaluation, and analysis of dynamic communities, has important academic research significance and socio-economic value.

Community detection is to identify the existing community structure from the complex network. As a collection of specific objects, the community has a significant node aggregation structure and a node distribution form with statistical characteristics [2], which provides the possibility for accurate dynamic community detection. At present, community detection algorithms can be roughly divided into graph segmentation-based method [3], random walk-based method, modularity-based method [4, 5], label propagation-based method [6], node centrality-based method [7], and neural network-based method. The existing researches on community detection are often based on the impact of static network structure on community division. For example, Bouguessa et al. used the covariance of links between nodes and interclass inertia to perform the initial division of the network and determined the maximum modular community structure by merging the initial groups in the iterative process, but this method was limited by the impact of different resolution parameters on the correctness of community division [8]. Cai et al. carried out multiobjective optimization of network model based on the evolutionary algorithm, but multiple iterations occupied a lot of computing resources [9]. Ni et al. proposed a detection structure for local overlapping communities, which improved the efficiency of local community detection [10]. However, there was a problem of large deviation of representative nodes, which often led to only the local optimal solution. The above community detection methods based on static network structure have a certain dependence on priori data, and due to the lack of real-time computing ability, it is limited by the influence of parameters on the detection results.

With the continuous expansion of the dataset scale, how to continuously reconstruct the node features according to the increase of data dimension and realize the dynamic detection of complex network communities is still a problem to be solved. For example, Moscato et al. proposed an online social network community detection algorithm based on game theory, but the mathematical statistical model of dynamic game based on individual behavior put forward high requirements for memory space, and there was the possibility of dimension disaster when solving [11]. In addition, with the development of graph neural network in recent years, it has more advantages in extracting node features and preserving graph structure, which has attracted some researchers to use the graph neural network to solve the problem of community detection. For example, Chen et al. regarded community detection as an extended node classification task, proposed a line graph neural network (LGNN) model, and designed the adjacency matrix based on polynomial function and nonbacktracking operators for community detection [12]. However, the graph storage method using an adjacency matrix needs to be traversed when counting elements, which has high time complexity. Luo et al. constructed a context path-based graph neural network (CP-GNN) by using the high-order relationship between nodes, which recursively embedded the high-order relationship between nodes into the node with an attention mechanism to distinguish the importance of different relationships [13]. Based on graph convolutional neural network (GCN) and label propagation technology, Wang et al. constructed a balanced label set to reveal the underlying community structure with topology and attribute information [14]. However, as weak supervised learning algorithms, the above two methods are relatively fragile to abnormal data and are difficult to define relevant parameters. The existing dynamic community detection methods based on the graph neural network overemphasize the ability to distinguish different graph structures and ignore the local expression ability of nodes, resulting in the oversmoothing problem [15, 16]. That is, the node feature representation in the same connected component tends to converge to the same value after multiple convolutions, making it difficult to distinguish nodes.

With the growing importance of network dynamic data detection under the development of information technology, traditional detection methods for dynamic communities in complex networks have limited the performance of dynamic community detection due to the emergence of node oversmoothing problems and the influence of a priori model parameters. To address these problems, a method for detecting dynamic communities in complex networks based on deep self-coding networks is proposed. Compared with the existing community detection methods based on the graph, the innovations of the proposed method are as follows:

1. An algorithm framework of encoding-decoding mechanism based on deep self-coding network is proposed, which realizes the re-evaluation of the features of the initial nodes, effectively solves the problem of node oversmoothing, and improves the accuracy of graph classification.
2. From the perspective of community detection task, the loss function related to community detection is defined. It ensures the update of parameters in the network model and improves the efficiency of community detection algorithm.

The following sections are arranged as follows: the second section defines the problems studied; the third section introduces the proposed dynamic community detection method based on deep self-coding network; in Section 4, experiments are designed to verify the performance of the proposed community detection method; the fifth section is the conclusion.

## 2. Problem Definition

Community detection refers to the discovery of densely connected subnetworks in the graph structure. Liu et al. defined the community as follows: (1) the nodes in the community are densely connected; (2) the nodes in different communities are sparsely connected [17]. The community division under a basic network is shown in Figure 1.

In a dynamic network, each timestamp *i* corresponds to the corresponding network structure *G*_*i*_=(*V*_*i*_, *E*_*i*_), where *V*_*i*_ and *E*_*i*_ represent the node set and edge set corresponding to timestamp *i*, respectively. It is necessary to obtain the basic community structure under each timestamp and sort it according to the time series 1,…, *t*. In order to extract and learn the network representation information comprehensively, the snapshot iteration method will be used to reflect the information of the dynamic network. Due to the large amount of data of the snapshot information, the time consumption of predicting the community based on the global snapshot iteration method is too high. Although it is reasonable and comprehensive, it is not efficient, so this method is abandoned; in addition, community prediction based on independent snapshot iteration has the same effect as dynamic network community detection. Although it is efficient, the dynamic time correlation is not strong, so it is impossible to predict the community. Therefore, the second-order snapshot iteration can ensure the rationality of dynamic information and reduce the time overhead to a certain extent. The community structure contains many key points with potential characteristics. Different matrices are used to define different parts of the data, such as links and contents. This method will re-embed the shared matrix composed of multiple information in the network at different times into the shared feature matrix, so as to improve the effect of community detection.

**Definition 1 .**

(dynamic community prediction). Given a series of snapshot sequences of graphs *G*_1_,…, *G*_*i*_,…, *G*_*t*_ with *n* × *n* adjacency matrix *P*_1_,…, *P*_*i*_,…, *P*_*t*_ and *n* × *d* content matrix *Q*_1_,…, *Q*_*i*_,…, *Q*_*t*_, a shared matrix *W*_1_,…, *W*_*i*_,…, *W*_*t*_ is formed to predict the network structure under future time *t*+Δ*t*.

For the community prediction of dynamic network, the network snapshot information needs to be iterated. When predicting the community structure under the time *t*+Δ*t*, the sharing matrices *W*_1_,…, *W*_*i*_,…, *W*_*t*+1_, *W*_*t*_ of previous snapshots need to be used to enhance the accuracy of prediction results.

## 3. Dynamic Community Detection Based on Deep Self-Coding Network

### 3.1. Node Feature Reconstruction Based on Encoding-Decoding Mechanism

In the graph convolution neural network, the node representation that captures the local structure and feature information of the graph will be fed to the global readout module to refine for graph-level representation learning. However, the graph-level representation ability and discrimination ability of traditional GCN are limited by over-refining and globalization, ignoring the preservation of local features, which will lead to the problem of oversmoothing. In order to alleviate these problems, an encoding-decoding mechanism is designed in the model to reconstruct the feature information of each node in the graph. The stack of multiple graph convolution layers is regarded as an encoder that encodes the node feature information into the potential vector space, and the decoder uses a simple two-layer perceptron to reconstruct the initial node feature from the encoded vector information. The encoding-decoding mechanism realizes the re-evaluation of the features of the initial node. Then, an additional local feature reconstruction loss is added after the decoder to assist the goal of graph classification and improve the accuracy of graph classification.

According to the model diagram shown in Figure 2, the encoder composed of K graph convolution layers aggregates local adjacent information at different structural levels. After the K-iteration of neighborhood aggregation, the output of the encoder extracts the local structure information and node feature information in the K-hop neighborhood. The encoder encodes the node feature of each node into an intermediate representation, and the decoder aims to map the encoded node representation to the reconstructed feature vector $\hat{Z}\in R$. From Figure 2, given the graph-level representation *k*_(*K*)*G*_ ∈ *R*^*do*^ of the readout module of the upper layer, the reconstructed features $\hat{\text{Z}}$ can be calculated according to the following formula:

(1) $$\begin{array}{c} \hat{Z}=\text{Dec}\left(\sum_{i=1}^{t-1}k_{v}^{\left(i\right)}\right). \end{array}$$

A two-layer perceptron is used as the decoder. It is worth mentioning that the encoding-decoding mechanism is different from the graph self-encoder model [18–20]. The decoder is to reconstruct the initial node features, rather than a task-specific classifier to recover the adjacency information of the graph.

### 3.2. Community Detection Loss Function

Referring to the LGNN model [21], this study defines the loss function for the community detection task. In the community detection task, the node label should follow the equivalent replacement invariant property of the community [22]; that is, the divided community is not affected by the specific meaning of a specific label. From the output of Section 3.1, the predicted probability ${\hat{a}}_{i}$ of the community to which each node belongs is obtained through Softmax. Let *A* represent the set of labels for all communities, and *A*_*i*_ represent the real probability of the community to which each node belongs. Therefore, the loss function is defined as follows:

(2) $$\begin{array}{c} S=\underset{\pi \in S_{A}}{\text{INF}}-\sum_{i\in R}\pi \left(a_{i}\right)\log\left({\hat{a}}_{i}\right), \end{array}$$

where INF represents the infimum of the function, *S*_*A*_ is the permutation and combination set of all communities *A*, and *π* is an permutation in *S*_*A*_. Assuming that *F*_1_ : *E*⟶*A* is the function mapping from the initial feature matrix *E* of the node to the real community *A*, $F_{1}:E⟶\hat{A}$ is the function mapping from the initial feature matrix *E* of the node to the model predicted community $\hat{A}$, and *t*_*i*_ represents the feature vector of each node in the matrix, then the final loss function formula can be obtained from the following formula:

(3) $$\begin{array}{c} S=\underset{\pi \in S_{A}}{\text{INF}}-\sum_{i\in R}F_{1}\left(\pi \left(x_{i}\right)\right)\log\left(F_{2}\left(\pi \left(x_{i}\right)\right)\right). \end{array}$$

The ultimate goal of the loss function is to take the minimum cross-entropy loss on all possible permutations, so as to update the parameters in the network model.

### 3.3. Self-Coding Learning Process

Stochastic gradient descent is used to optimize the loss function. Specifically, the parameters *γ*={*M*, *M*^*∗*^, *u*, *u*^*∗*^} of the algorithm framework are updated in each iteration according to the following contents:

(4) $$\begin{array}{c} \left\{\begin{array}{c} M_{ij}=M_{ij}-\beta \frac{\partial }{\partial M_{ij}}S_{\gamma }\left(\hat{T},{\hat{T}}^{*}\right),\\ M_{ij}^{*}=M_{ij}^{*}-\beta \frac{\partial }{\partial M_{ij}^{*}}S_{\gamma }\left(\hat{T},{\hat{T}}^{*}\right),\\ u_{ij}=u_{ij}-\beta \frac{\partial }{\partial u_{ij}}S_{\gamma }\left(\hat{T},{\hat{T}}^{*}\right),\\ u_{ij}^{*}=u_{ij}^{*}-\beta \frac{\partial }{\partial u_{ij}^{*}}S_{\gamma }\left(\hat{T},{\hat{T}}^{*}\right), \end{array}\right) \end{array}$$

where *β* is the learning rate and (*·*)^*∗*^ indicates reconstruction. Due to the similarity of the inference processing between *M*, *u* and *M*^*∗*^, *u*^*∗*^, only the inference of the update rule of parameter *M*, *u* is shown as follows:

(5) $$\begin{array}{c} \frac{\partial }{\partial M_{ij}}S_{\gamma }\left(\hat{T},{\hat{T}}^{*}\right)=\sum_{i=1}^{N}\frac{\partial }{\partial M_{ij}}S_{\gamma }\left(t_{i},g\left(\phi \left(t_{i}\right)\right)\right)\\ =\sum_{i=1}^{N}\frac{\partial }{\partial k_{i}^{n}}S_{\gamma }\left(t_{i},g\left(\phi \left(t_{i}\right)\right)\right)\frac{\partial }{\partial M_{ij}}k_{i}^{n}\\ =\sum_{i=1}^{N}\alpha_{i}T_{i}^{\tau }, \end{array}$$

where *k*_*i*_=*M·z*_*i*_+*u*, and *α*_*i*_=(*∂*/*∂k*_*i*_^*n*^)*S*_*γ*_(*t*_*i*_, *g*(*ϕ*(*t*_*i*_))) represents the characterization term of each node for the overall error. In order to measure the difference between the input data $\hat{T}$ and ${\hat{T}}^{*}$, the *α*_*i*_ in the encoder is written as follows:

(6) $$\begin{array}{c} \alpha_{i}=\frac{\partial }{\partial k_{i}^{n}}S_{\gamma }\left(t_{i},g\left(\phi \left(t_{i}\right)\right)\right)\\ =-\sum_{i=1}^{N}\frac{\partial }{\partial k_{i}^{n}}S_{\gamma }\left({\hat{T}}_{ij},{\hat{T}}_{ij}^{*}\right)\cdot \text{Relu}{}^{\prime }\left(k_{i}^{n}\right), \end{array}$$

where Relu(*·*) is the linear rectification function and Relu′(*·*) is the derivative of Relu(*·*). In the decoder, *v*_*i*_=*M*^*∗*^*·k*+*u*, and the characterization item *α*_*i*_^*∗*^ is as follows:

(7) $$\begin{array}{c} \alpha_{i}^{*}=\left(\sum_{i=1}^{r}M_{ij}^{*}\cdot \alpha_{i}\right)\cdot \text{Tanh}{}^{\prime }\left(k_{i}^{n}\right), \end{array}$$

where Tanh(·) is activation function and Tanh′(·) is the derivative of Tanh(·).

### 3.4. Algorithm Framework Description

Deep learning has excellent data learning ability and representation ability. Through training multilayer neural network, the representation information learned in each layer is used as input data and input into the next neural layer. Therefore, a deep automatic encoder with a multilayer automatic encoder is constructed and trained in the first layer of automatic encoder by reconstructing the input matrix $\hat{Y}$. Then, the best potential representation *K*^1^ ∈ *R*^*r*^1^×*N*^ is obtained. Finally, the next automatic encoding layer is trained by reconstructing *K*^1^ from the above automatic encoder, and a new potential representation *K*^2^ ∈ *R*^*r*^2^×*N*^ is obtained. Then, the potential feature matrix output by the hidden layer is reinput to the decoding layer with the same layer number as the encoding layer. The encoding and decoding layers have a symmetrical structure.

By continuously optimizing the learning parameters, remapping the compressed matrix to the size of the original matrix, learning the community structure information under multiple timestamps, and analyzing it, the evolution trend of the future community can be obtained, so as to predict the community network structure under timestamps *t*+Δ*t*. The workflow of this algorithm framework is shown in Figure 3. By fusing the node topology and text information under multiple timestamps, combined with time analysis, the feature information containing community evolution trend is formed, and the potential information is extracted through representation learning.

Because the extracted potential representation contains both the structure information of the current community and the evolution information of the community, it can be used to predict the evolution trend of the future community. The algorithm framework is shown in Algorithm 1. Steps 1 to 4 are to fuse the adjacency matrix *P* and content matrix *Q* under multiple time snapshots, initialize the network, and set the number of iterations *ζ* and the depth *L* of the self-coding network. Steps 5 to 12 are to extract the dynamic network information by using the deep self-coding network. After the two parts of encoding and decoding in the self-coding network, steps 13 and 14 are to reconstruct the network information through the learned potential representation. These steps can predict the future community structure and carry out clustering operation, so as to obtain the community structure of dynamic network.

## 4. Experiment and Analysis

The hardware configuration of the experiment is as follows: 8 GB memory, i5-4200H dual-core processor, and Windows 10 operating system. The compiler used for algorithm development is VisualStudio Code, the code is written in Python language, its version is 3.6.2, and the Pytoch framework is used. In order to measure the convergence and detection accuracy of the proposed algorithm, the line graph neural network (LGNN) algorithm proposed in reference [12], the context path-based graph neural network (CP-GNN) algorithm proposed in reference [13], and the algorithm based on graph convolution network (GCN) and label propagation technology proposed in reference [14] are selected as a comparison to verify the performance of the proposed model. The description of each algorithm is listed in Table 1.

### 4.1. Experimental Dataset

Two classical complex networks such as Karate Club network (Karate) [23] and American Football League network (Football) [24] are used for experiments to verify and analyze the community division performance of different algorithms. The following is a brief description of each dataset:

1. *Karate Club*. This network depicts the interpersonal relationship between members of a karate club in an American University. The members of the club are divided into two factions due to differences on a certain issue, as shown in Figure 4.
2. *Football*. This dataset is the game relationship between football teams of different universities in the United States in the 2000 season. The node represents the participating football teams, while the side indicates that the two teams have played this season.

The statistics of each dataset are listed in Table 2.

### 4.2. Experimental Evaluation Index and Convergence Analysis

#### 4.2.1. Experimental Evaluation Index

The evaluation indexes used in this experiment are accuracy, F1-score, NMI, and modularity.

(1) *Accuracy*. It is a common evaluation index for node classification. It evaluates the correctly predicted sample ratio.
(2) *F1-score*. It is applicable to the evaluation index of classification task. It takes into account the proportion of samples predicted to be true that are actually true, and the proportion of samples actually true that are predicted true. The macro-F1 index is used in the experiment. First, the F1-scores of precision and recall of each data sample are calculated respectively, and then all results are averaged to obtain the final result.
(3) *NMI*. It refers to normalized mutual information. It measures the similarity between two clusters, and it is an important evaluation index for community detection. The higher the NMI score, the better the detection effect. Supposing that *Z*_true_ is the real cluster and *Z*_pred_ is the cluster prediction result, then the formula is defined as follows:
  (8) $$\begin{array}{c} \left\{\begin{array}{c} \text{NMI}\left(Z_{\mathrm{pred}};Z_{\mathrm{true}}\right)=2\frac{I\left(Z_{\mathrm{pred}};Z_{\mathrm{true}}\right)}{H\left(Z_{\mathrm{pred}}\right)+H\left(Z_{\mathrm{true}}\right)},\\ H\left(Z_{\mathrm{pred}}\right)=-\sum_{\hat{z}}p\left(\hat{z}\right)\log\left(p\left(\hat{z}\right)\right),\\ I\left(Z_{\mathrm{pred}};Z_{\mathrm{true}}\right)=\sum_{\hat{z}}\sum_{z}p\left(\hat{z},z\right)\log\left(\frac{p\left(\hat{z},z\right)}{p\left(\hat{z}\right)p\left(z\right)}\right). \end{array}\right) \end{array}$$
(4) *Modularity*. It is used to evaluate the quality of the detected community. It is defined as follows:
  (9) $$\begin{array}{c} M_{o\;du}=\frac{1}{2}\sum_{i\neq j}\left(P_{ij}-\frac{p_{i}p_{j}}{2y}I\left(b_{i},b_{j}\right)\right), \end{array}$$

where *P*_*ij*_ is the element in the graph adjacency matrix, *y* is the number of edges, *p*_*i*_=∑_*j*_*P*_*ij*_ is the sum of degrees of the *i*-th node, and *b*_*i*_ is the community of the *i*th node. If *b*_*i*_=*b*_*j*_, then *I*(*b*_*i*_, *b*_*j*_)=1; otherwise, *I*(*b*_*i*_, *b*_*j*_)=0. The higher the modularity result, the more edges in the community and the fewer edges between communities.

#### 4.2.2. Convergence Analysis

The convergence of the proposed model will be analyzed on the Karate Club and Football datasets. Since each iteration of the algorithm mainly updates the relationship tightness between nodes, the convergence of the algorithm is analyzed by comparing the difference of the relationship matrix before and after updating with the number of iterations. Based on the trusted nearest neighbor graph, the indirect tightness of non-nearest neighbor nodes is obtained through similarity propagation. In addition, considering the inheritance and update of information in the iterative process of the algorithm, the similarity update rule between two sections *i* and *j* is defined as follows:

(10) $$\begin{array}{c} X_{s\_ij}^{t}=\lambda {\tilde{X}}_{s\_i}{\left({\tilde{X}}_{s\_j}\right)}^{T}+\left(1-\lambda \right)X_{s\_ij}^{t-1}. \end{array}$$

The first item is the nonzero element in the indirect tightness ${\tilde{X}}_{s\_i}$ of the two nodes, that is, the highly trusted nearest neighbor node of node *i*. In the above iterative process, not only the connection information before the update of the two nodes is retained, but also the indirect tightness of the node pair is introduced by its common nearest neighbor, and the parameter *λ* controls the proportion of the two in the similarity update process. After several iterations, the tightness between nodes tends to be stable, and then, the square error ‖*X*_*s*_^*t*+1^ − *X*_*s*_^*t*^‖_*F*_ of the similarity matrix before and after the iteration can be recorded based on the updated node similarity matrix.  Figure 5 shows the change curves of the square error with the number of iterations in the two datasets.

It can be seen from the figure that after about 13 iterative updates, the tightness between nodes tends to be stable, which verifies the convergence of the algorithm.

### 4.3. Experimental Results

#### 4.3.1. Comparison and Analysis of Test Results

The community detection results are listed in Tables 3 and 4. On the experimental results of Karate Club dataset (Table 3), the performance of the proposed model is significantly better than all other methods in all evaluation indexes.

Because the LGNN algorithm [12] adopts the graph storage method of adjacency matrix, it needs to traverse when counting elements, which has high time complexity and further affects the detection accuracy and performance. The CP-GNN algorithm [13] and GCN algorithm [14] due to the relative vulnerability of weak supervised learning algorithm to abnormal data and the oversmoothing problem of the algorithm itself, the accuracy of clustering detection results has been affected to a certain extent. It can be seen from Table 3 that the proposed model is relatively optimal in the experimental results of Karate Club dataset, especially in the NMI index. Compared with the LGNN algorithm [12] model, the NMI is increased by 9.98%. Compared with the CP-GNN algorithm [13] model, the NMI is improved by 6.60%. Compared with the GCN algorithm [14] model, the NMI is improved by 6.36%. In addition, the accuracy and F1-score of the proposed model show that the proposed method can detect the community more accurately. Compared with the methods with oversmoothing problem (such as the GCN algorithm [14]), the proposed model uses an encoding-decoding mechanism to reconstruct the feature information of each node in the graph, which can explain its superior performance. It can be seen from the results of Karate Club dataset that it is very important to consider the reconstruction of node features in the process of algorithm execution.

The superiority of the proposed model can also be observed in the experimental results of Football dataset (Table 4). However, the NMI of LGNN algorithm [12] is similar to that of the proposed model. One possible reason is that the LGNN algorithm [12] uses a so-called “nonbacktracking” operator, which can well preserve the spatial node information across multiple steps. In contrast, the proposed model may have slight data loss in the reconstruction of data nodes by using the encoding-decoding mechanism, so it has no significant advantage in the NMI index. Although the other two algorithms (CP-GNN algorithm [13] and GCN algorithm [14]) can better retain the long-term time features, if more time map data are convoluted, then the embedded features may become too smooth, so that the distance between all nodes becomes close. Therefore, it cannot accurately detect the community, resulting in a slight weakness in the evaluation index. In the modularity index, the proposed model performs best. Compared with the LGNN algorithm [12] model, the modularity is improved by 26.42%. Compared with the CP-GNN algorithm [13] model, the modularity is improved by 19.29%. Compared with the GCN algorithm [14] model, the modularity is improved by 15.19%.

#### 4.3.2. Results and Analysis of Label Rate Impact

In order to observe the influence of the training label rate on the experimental results, the experiment selects accuracy and NMI indexes to evaluate all methods on the Football dataset. In this experiment, the training label rates are 10%, 20%, 30%, 50%, and 70%, respectively. The experimental results are shown in Figures 6 and 7.

As shown in Figure 6, in terms of accuracy index, with the increase of training label rate, the model performance of all methods is gradually improving. However, the accuracy index of LGNN algorithm [12] is not ideal. The possible reason is that the LGNN model affects the detection accuracy of the model in the process of traversing elements through the graph storage method of adjacency matrix. When the training label rate is 70%, the accuracy index of the proposed model is improved by 6.45% compared with the LGNN algorithm [12]. Compared with the CP-GNN algorithm [13], accuracy is improved by 5.32%. Compared with the GCN algorithm [14], accuracy is improved by 3.13%. Experimental results show that the proposed algorithm has higher execution accuracy. Based on the graph convolution neural network algorithm, the inherent oversmoothing problem of the algorithm is overcome through the encoding-decoding mechanism, so as to improve the detection efficiency and accuracy.

Figure 7 shows that when the training label rate increases from 10% to 70%, the F1-score index of all algorithms gradually increases. Because the typical graph convolution neural network method belongs to the weak supervised learning algorithm, it is relatively fragile to abnormal data and difficult to define relevant parameters. Therefore, with the expansion of the scale of training label rate, the F1-score index continues to slow down. Due to the setting of community detection loss function, the proposed model will update the parameters in the network model during the detection process, so it has better performance. When the training label rate is 70%, the F1-score index of the proposed model is 17.33% higher than that of LGNN algorithm [12]. Compared with the CP-GNN algorithm [13], F1-score is increased by 16.56%. Compared with the GCN algorithm [14], F1-score is improved by 7.32%.

## 5. Conclusion

Aiming at the problems that the traditional community detection methods are greatly affected by priori parameters, a complex network dynamic community detection method based on deep self-coding network is proposed. The basic ideas are as follows: ① algorithm framework based on encoding-decoding mechanism; ② local feature reconstruction based on decoding results; ③ establishment of community detection loss function. Experimental results show that compared with the original method, the proposed algorithm has detection accuracy and realizes the effective detection of complex network community structure. At present, the proposed model can only be tested on graphs of moderate size, and it has been proved that the proposed model is not enough for large-scale graphs in terms of architecture and training algorithm. The main research direction in the next step is how to achieve the correct compromise between performance, computational complexity, memory consumption, training, and reasoning time, and finally improve the performance.

## Figures and Tables

**Figure 1:** Community structures in networks.

**Figure 2:** A three-layer model for graph classification.

**Figure 3:** Algorithm framework.

**Figure 4:** Karate Club network.

**Figure 5:** Convergence analysis.

**Figure 6:** Experimental results of accuracy index with different training label rates.

**Figure 7:** Experimental results of F1-score with different training label rates.

**Algorithm 1:** Community detection algorithm.

**Table 1:** Dynamic community detection algorithms.

Algorithm	Description
Line graph neural network (LGNN) [12]	The high-level graph algorithm is realized by sparse matrix multiplication and message passing
Context path-based graph neural network (CP-GNN) [13]	The nodes of an input graph are classified by weak supervision
Graph convolution network (GCN) algorithm [14]	Local parameters are shared and the receptive field is proportional to the number of layers
The proposed model	The temporal information is effectively combined to transition oversmooth process

**Table 2:** Description of dataset.

Network	Node	Edge	Community
Karate Club	34	78	2
Football	115	613	12

**Table 3:** Community detection results for different algorithms on the Karate Club dataset (%).

Algorithms	Accuracy	F1-score	NMI	Modularity
LGNN [12]	89.3	92.3	85.2	63.7
CP-GNN [13]	94.1	92.1	87.9	62.3
GCN [14]	95.4	94.8	88.1	64.9
The proposed method	96.6	95.2	93.7	65.2

**Table 4:** Community detection results for different algorithms on the Football dataset (%).

Algorithms	Accuracy	F1-score	NMI	Modularity
LGNN [12]	60.1	60.9	49.7	31.8
CP-GNN [13]	58.9	61.2	43.6	33.7
GCN [14]	61.4	64.8	44.7	34.9
The proposed method	64.2	67.0	50.3	40.2

## Data Availability

The data used to support the findings of this study are included within the article.

## References

[1] Liu W., Gong M., Tang Z., Qin A., Sheng K., Xu M. (2021). Locality preserving dense graph convolutional networks with graph context-aware node representations. *Neural Networks*.

[2] Kichikawa Y., Iyetomi H., Iino T., Inoue H. (2019). Community structure based on circular flow in a large-scale transaction network. *Applied Network Science*.

[3] Qiu J., Peng J., Zhai Y. Network community detection based on spectral clustering.

[4] Tang L., Wang X., Liu H. (2012). Community detection via heterogeneous interaction analysis. *Data Mining and Knowledge Discovery*.

[5] Tang L., Wang X., Liu H. Uncovering groups via heterogeneous interaction analysis.

[6] Chen J., Liu M., Liu X. (2019). Research on of overlapping community detection algorithm based on tag influence. *Cluster Computing*.

[7] Ma T., Liu Q., Cao J., Tian Y., Al-Dhelaan A., Al-Rodhaan M. (2020). LGIEM: global and local node influence based community detection. *Future Generation Computer Systems*.

[8] Bouguessa M., Missaoui R., Talbi M. A novel approach for detecting community structure in network.

[9] Cai Q., Ma L., Gong M., Tian D. (2016). A survey on network community detection based on evolutionary computation. *International Journal of Bio-Inspired Computation*.

[10] Ni L., Luo W., Zhu W., Hua B. (2020). Local overlapping community detection. *ACM Transactions on Knowledge Discovery from Data*.

[11] Moscato V., Picariello A., Sperlí G. (2019). Community detection based on game theory. *Engineering Applications of Artificial Intelligence*.

[12] Chen Z., Li X., Bruna J. Supervised community detection with line graph NeuralNetworks.

[13] Luo L., Fang Y., Cao X., Zhang X., Zhang W. Detecting communities from heterogeneous graphs: a context path-based graph neural network model.

[14] Wang X., Li J., Yang L., Mi H., Yu J. Y. (2021). Weakly-supervised learning for community detection based on graph convolution in attributed networks. *International Journal of Machine Learning and Cybernetics*.

[15] Chen D., Lin Y., Li W., Li P., Zhou J., Sun X. Measuring and relieving the over-smoothing problem for graph neural networks from the topological view.

[16] Protas E., Bratti J. D., Gaya J. F. O., Drews P., Botelho S. S. C. (2019). Visualization methods for image transformation convolutional neural networks. *IEEE Transactions on Neural Networks and Learning Systems*.

[17] Liu F., Xue S., Wu J. Deep learning for community detection: progress, challenges and opportunities.

[18] Vercheval N., De Bie H., Pižurica A. Variational auto-encoders without graph coarsening for fine mesh learning.

[19] Wang Z., Wang L., Liu S., Wei G. (2018). Encoding-Decoding-Based control and filtering of networked systems: insights, developments and opportunities. *IEEE/CAA Journal of Automatica Sinica*.

[20] Li T., Xie L. (2012). Distributed coordination of multi-agent systems with quantized-observer based encoding-decoding. *IEEE Transactions on Automatic Control*.

[21] Xiong X., Ozbay K., Jin L., Feng C. (2020). Dynamic origin-destination matrix prediction with line graph neural networks and kalman filter. *Transportation Research Record: Journal of the Transportation Research Board*.

[22] Guo K., Huang X., Wu L., Chen Y. (2022). Local community detection algorithm based on local modularity density. *Applied Intelligence*.

[23] Zachary W. W. (1977). An information flow model for conflict and fission in small groups. *Journal of Anthropological Research*.

[24] Newman M. E. J. (2006). Modularity and community structure in networks. *Proceedings of the National Academy of Sciences*.

